# Activation of the AMP-Activated Protein Kinase (AMPK) by Nitrated Lipids in Endothelial Cells

This article has been retracted.

**DOI:** 10.1371/journal.pone.0031056

**Published:** 2012-02-17

**Authors:** Yong Wu, Yunzhou Dong, Ping Song, Ming-Hui Zou

**Affiliations:** 1 Section of Molecular Medicine, Department of Medicine, Department of Biochemistry and Molecular Biology, University of Oklahoma Health Sciences Center, Oklahoma City, Oklahoma, United States of America; 2 Department of Biochemistry, University of California, Riverside, Riverside, California, United States of America; University of Hong Kong, China

## Abstract

The AMP-activated protein kinase (AMPK) is an important regulator of endothelial metabolic and functional homeostasis. Here, we examined the regulation of AMPK by nitrated oleic acid (OA-NO_2_) and investigated the implications in endothelial function. Treatment of bovine aortic endothelial cells (BAECs) with OA-NO_2_ induced a significant increase in both AMPK-Thr172 phosphorylation and AMPK activity as well as upregulation of heme oxygenase (HO)-1 and hypoxia-inducible factor (HIF)-1α. Pharmacologic inhibition or genetic ablation of HO-1 or HIF-1α abolished OA-NO_2_-induced AMPK phosphorylation. OA-NO_2_ induced a dramatic increase in extracellular signal-regulated kinase (ERK)1/2 phosphorylation that was abrogated by the HO-1 inhibitor, zinc deuteroporphyrin IX 2,4-bis-ethylene glycol (ZnBG). Inhibition of ERK1/2 using UO126 or PD98059 reduced but did not abolish OA-NO_2_-induced HIF-1α upregulation, suggesting that OA-NO_2_/HO-1-initiated HIF-1α induction is partially dependent on ERK1/2 activity. In addition, OA-NO_2_ enhanced endothelial intracellular Ca^2+^, an effect that was inhibited by the HIF-1α inhibitor, YC-1, and by HIF-1α siRNA. These results implicate the involvement of HIF-1α. Experiments using the Ca^2+^/calmodulin-dependent protein kinase kinase (CaMKK) inhibitor STO-609, the selective CaMKII inhibitor KN-93, and an isoform-specific siRNA demonstrated that OA-NO_2_-induced AMPK phosphorylation was dependent on CaMKKβ. Together, these results demonstrate that OA-NO_2_ activates AMPK in endothelial cells via an HO-1–dependent mechanism that increases HIF-1α protein expression and Ca^2+^/CaMKKβ activation.

## Introduction

Accumulating evidence indicates that reactive nitrogen species (RNS), which are inflammatory oxidants, mediate diverse physiologic and pathologic processes in cardiovascular, pulmonary, and neurodegenerative diseases [1]. RNS, such as peroxynitrite (ONOO^−^), nitrogen-dioxide radical, and nitronium ion, which are formed from nitric oxide (NO), are important factors in complications of obesity and diabetes [2]. RNS react with unsaturated fatty acids to form relatively stable nitrated products (nitroalkene derivatives), including the abundant and clinically important nitrated oleic and linoleic acids [3]. Although this process occurs via various mechanisms, the common denominator is a proclivity for homolytic addition of nitrogen dioxide (•NO_2_) to the double bond, yielding an array of regio- and stereoisomers [4]. Nitrated unsaturated fatty acids (NO_2_-UFAs) represent a convergence of lipid and NO signaling and have emerged as a novel class of endogenously produced vascular signaling molecules [5]. The beneficial effects of NO_2_-UFAs include cGMP-dependent vessel relaxation, inhibition of inflammatory cell function, adaptive and anti-inflammatory cell responses, induction of heme oxygenase-1 (HO-1) expression, inhibition of nuclear factor (NF)-κB, and activation of peroxisome proliferator activated receptor (PPAR) and Keap1/Nrf2 [6].

Plasma free and esterified nitrated oleic acid (OA-NO_2_) concentrations have been reported to be 619±52 and 302±369 nM, respectively, and these levels are approximately 50% greater than the level of nitrated linoleic acid (LNO_2_). The combined blood levels of the free and esterified fatty acid derivatives exceeds 1 µM [4]. The plasma levels of NO_2_-UFA derivatives in hyperlipidemic patients are elevated relative to levels in normolipidemic subjects [7]. In addition, an increase in oxidative stress in hypercholesterolemia [8] may contribute to the formation of nitrated species in the vascular wall [9]. Thus, nitrated lipids in the plasma can be used as an indicator of the chain-breaking antioxidant role of NO in lipid oxidation [10] and/or provide a footprint for the presence of oxidants/nitrating agents in the vascular system. We postulate that the presence of these nitrated products *in vivo* promote cardiovascular homeostasis and compensate for impaired vascular endothelial function in the context of dyslipidemia, obesity, and diabetes. The molecular target(s) and mechanisms underlying the vascular-protective and anti-inflammatory effects of NO_2_-UFAs remain poorly defined.

The serine/threonine kinase, AMP-activated protein kinase (AMPK), is a member of the Snf1/AMPK protein kinase family that is found in all eukaryotes [11]. This kinase is thought to act as a cellular energy sensor by stimulating ATP-producing catabolic pathways and inhibiting ATP-consuming anabolic pathways [12]. AMPK is comprised of three subunits: a catalytic α-subunit and regulatory β- and γ-subunits. Activation of AMPK requires the phosphorylation of Thr172 in the activation loop of the α-subunit by an upstream AMPK kinase (AMPKK) [13]. Interestingly, the first AMPKK to be identified was LKB1, a tumor suppressor that is mutated in humans with Peutz-Jegher syndrome [14]. Patients with this syndrome have an increased risk of developing carcinomas of the colon, stomach, and pancreas. Recently, calcium (Ca^2+^) calmodulin-dependent kinase kinase (CaMKK) [15] was identified as an upstream AMPKK. CaMKK is activated by a rise in intracellular Ca^2+^ concentrations ([Ca^2+^]_i_), and this kinase phosphorylates and activates AMPK in an AMP-independent manner [15]. Therefore, in addition to responding to an increase in the AMP-to-ATP ratio, AMPK may also be activated by a rise in [Ca^2+^]_i_ in response to nutrients, drugs, or physiological stimuli. While the AMPK pathway is traditionally thought to be a regulator of metabolism, recent studies have demonstrated that AMPK may also act to maintain endothelial function [16]. AMPK exerts pleiotropic effects that are believed to be beneficial for endothelial function. These effects, which are ultimately anti-atherogenic, include induction of the endothelial nitric oxide synthase (eNOS)/NO pathway and result in an increase in NO bioavailability, suppression of endothelial ROS production following exposure to deleterious stimuli, such as hyperglycemia or high free fatty acids (FFAs), and modulation of vascular tone (see review [16]). AMPK also possesses anti-apoptotic and anti-inflammatory activities [17].

Since many of the metabolic changes and endothelial-protective effects attributable to NO_2_-UFAs are similar to those observed in response to AMPK activation, we hypothesized that AMPK activation is an important mediator of NO_2_-UFA activity. As such, AMPK activation may explain the pleiotropic beneficial effects of NO_2_-UFAs on the cardiovascular system in obesity and diabetes. Whether NO_2_-UFAs activate AMPK and, if so, by what mechanism(s) has yet to be determined. In the present study, we examined the effects of NO_2_-UFAs on the AMPK upstream kinases, specifically LKB1 and CaMKKβ. We also investigated whether NO_2_-UFAs modulate the eNOS/NO pathway, which is known to be an indicator of endothelial function and an important property of AMPK in cardiovasculature. We report that treatment with NO_2_-UFAs induces CaMKKβ-dependent AMPK activation through an HO-1/HIF-1α/Ca^2+^ pathway *in vitro* and show that NO_2_-UFAs promote p-eNOS and NO production via activation of the AMPK pathway in endothelial cells.

## Results

### OA-NO_2_ induces HO-1 protein and AMPK phosphorylation/activation in bovine aortic endothelial cells (BAECs)

To investigate activation of AMPK by OA-NO_2_ in endothelial cells, we treated confluent BAECs with different concentrations of OA-NO_2_ for 2–16 h. AMPK activation was indirectly assessed by western blot analysis of AMPK Thr172 phosphorylation, which is essential for AMPK activity [18]. As shown in Figure 1A and 1B, incubation of BAECs with OA-NO_2_ (0.5–2.5 µM for 16 h, or 2.5 µM for 2–16 h) resulted in a dose- and time-dependent increase in AMPKα phosphorylation at Thr172. AMPK Thr172 phosphorylation in BAECs gradually increased beginning 6 h after incubation with 2.5 µM OA-NO_2_ and reached peak levels after 16 h. This increased AMPK phosphorylation was associated with elevated AMPK activity, as measured by the SAMS peptide assay (Figure 1C). OA-NO_2_ treatment did not alter total AMPK levels, suggesting that OA-NO_2_-induced phosphorylation of AMPK was not due to altered expression of these proteins. Since OA-NO_2_ activated AMPK in both BAECs and human umbilical vein endothelial cells (HUVECs) at similar potencies, we performed the majority of our experiments with BAECs.

**Figure 1:** Induction of HO-1 protein and AMPK activation by OA-NO_2_. **A**) BAECs were incubated with OA-NO_2_ at the indicated concentrations or with BSA (vehicle) for 16 h, and western blot analysis was performed as described in Materials and Methods to detect HO-1 protein expression and AMPK phosphorylation at Thr172. The blot is representative of those obtained from three separate experiments. Corresponding densitometric analyses of phosphorylated AMPK and ACC are shown. *p<0.05 *vs.* control. **B**) BAECs were incubated with 2.5 µM OA-NO_2_ for the indicated times, and western blotting was performed as above. The blot is representative of three blots obtained from three separate experiments. *p<0.05 *vs.* corresponding control. **C**) Confluent BAECs were exposed to vehicle or OA-NO2 (2.5 µM) for 16 h. AMPKα was immunoprecipitated from cell lysates (1 mg) with a specific antibody. AMPK activity was assayed by ^32^P-ATP incorporation into the SAMS peptide. *p<0.05 *vs.* control. **D**) BAECs were incubated with the indicated concentrations of OA for 16 h. Western blotting was performed as described in Materials and Methods. **E**) BAECs were infected with Ad-DN-AMPK (MOI = 50) or Ad-GFP (control). Infected and non-infected cells were treated with 2.5 µM OA-NO_2_ for 16 h. AICAR and metformin were used as positive controls. The blot is representative of three blots obtained from three separate experiments.

The changes in AMPK phosphorylation were mirrored by changes in HO-1 protein expression, as evaluated by western blot analysis. Exposure of BAECs to a range of OA-NO_2_ concentrations resulted in an upregulation of HO-1 that was initially observed at 4 h with peak induction at 16 h. HO-1 induction and AMPK activation were specifically due to the nitroalkene moiety of OA-NO_2_, because oleic acid (OA) did not induce HO-1 protein expression or AMPK phosphorylation (Figure 1D). At a concentration of 2.5 µM, OA-NO_2_ potently activated AMPK and induced HO-1 expression without causing cellular toxicity. On the basis of these results, we chose to stimulate BAECs with 2.5 µM OA-NO_2_ for 16 h in subsequent experiments.

To determine whether OA-NO_2_-induced HO-1 expression was mediated by AMPK, we used an adenovirus encoding a dominant-negative mutant form of AMPKα (Ad-DN-AMPK) to suppress AMPK activity. AICAR (5-aminoimidazole-4-carboxamide-1-β-D-ribofuranoside) and metformin, two well characterized AMPK activators, were used as positive controls for AMPK phosphorylation. OA-NO_2_ significantly elevated AMPK phosphorylation (Figure 1E). As expected, Ad-DN-AMPK effectively suppressed AMPK phosphorylation but failed to abolish HO-1 induction by OA-NO_2_, suggesting that AMPK does not act upstream of HO-1 production in this system.

### Activation of AMPK by OA-NO_2_ does not require LKB1

Two recent studies [14], [19] showed that LKB1 acts as an upstream AMPK kinase. To evaluate the role of LKB1 in OA-NO_2_-induced AMPK activation, we investigated whether OA-NO_2_ altered LKB1 Ser 428 phosphorylation, which is essential for LKB1 activity and LKB1-dependent AMPK activation. As shown in Figure 2A, OA-NO_2_ did not alter the levels of LKB1 Ser428 phosphorylation.

**Figure 2:** Activation of AMPK by OA-NO_2_ does not require LKB1. **A**) Phosphorylation of LKB1 Ser428 was not affected by OA-NO_2_ in BAECs. Confluent BAECs were exposed to 2.5 µM OA-NO_2_ for 16 h, and phosphorylated LKB1-Ser428 was detected by a phospho-specific antibody in western blots. The blot is a representative of three blots obtained from three independent experiments. *Lower panels*: summary data (*n* = 3). **B**) LKB1 is not required for AMPK activation by OA-NO_2_. Confluent LKB1-deficient Hela-S3 cells were exposed to 2.5 µM OA-NO_2_ for 16 h, and then AMPK and ACC phosphorylation were assayed as described in Materials and Methods. The blot is representative of three blots obtained from three independent experiments. *Lower panels*: summary data (*p<0.05 *vs.* control; *n* = 3). **C**) LKB1 siRNA did not abolish OA-NO_2_-stimulated AMPK activation in HUVECs. HUVECs were incubated with LKB1-specific siRNA or control siRNA for 48 h and then treated with OA-NO_2_ or vehicle for 16 h. After treatment, cell lysates were analyzed for LKB1 protein levels and AMPK phosphorylation at Thr172. *Lower panels*: summary data (*p<0.05 *vs.* control; *n* = 3).

We next determined whether OA-NO_2_ activated AMPK in Hela-S3 cells, an LKB1-deficient cell line. Similar to the results obtained in BAECs, OA-NO_2_ (2.5 µM) induced AMPK phosphorylation on Thr172 in Hela-S3 cells (∼3-fold, *p*<0.05; Figure 2B). In parallel with AMPK phosphorylation, OA-NO_2_ dramatically increased phosphorylation of the known AMPK substrate, acetyl-CoA carboxylase (ACC), at Ser79 (∼2.4-fold, *p*<0.05), providing an additional indication that AMPK was activated in the absence of LKB1. To further explore the role of LKB1, we investigated the effect of siRNA-mediated LKB1 downregulation on AMPK activation induced by OA-NO_2_. As shown in Figure 2C, OA-NO_2_-induced AMPK phosphorylation was not significantly altered in cells pre-treated with LKB1 siRNA. The suppression of LKB1 protein expression by LKB1 siRNA (∼60%) was confirmed by western analysis. Taken together, these results strongly suggest that OA-NO_2_-induced phosphorylation of AMPK Thr172 is independent of its upstream kinase, LKB1.

### Induction of HIF-1α by OA-NO_2_ is dependent on HO-1

Hypoxia-inducible factor (HIF)-1 is a dimeric protein complex that plays an integral role in the body's response to hypoxia [20]. Like AMPK, HIF-1 is one of the primary genes involved in the homeostatic process that leads to increased vascularization in hypoxic areas, such as those within localized ischemia and in tumors [20]. HIF-1 and AMPK represent two main cellular pathways involved in coping with hypoxic stress and protecting cells against energy depletion and tissue reperfusion injury in times of metabolic crisis [21]. In addition, both HIF-1 and HO-1 are associated with ferrous iron metabolism [21]. Given that OA-NO_2_ induced both HO-1 expression and AMPK activation, we determined whether OA-NO_2_ also influenced HIF-1 expression. As predicted, OA-NO_2_ induced an increase in HIF-1α in HUVECs with a time course similar to OA-NO_2_-induced HO-1 expression and AMPK phosphorylation (Figure 3A). To explore the potential involvement of HO-1 in OA-NO_2_-induced HIF-1α expression, we pre-treated cells with the selective HO inhibitor zinc deuteroporphyrin IX 2,4-bis-ethylene glycol (ZnBG) and HO-1-specific siRNA. As shown in Figure 3A and B, ZnBG and HO-1 siRNA treatment abrogated the induction of HIF-1α protein expression and AMPK phosphorylation by OA-NO_2_, suggesting that OA-NO_2_ acts through the induction of HO-1 to increase HIF-1α expression and subsequently activate AMPK. The efficacy of the HO-1 siRNA in the downregulation of HO-1 expression was confirmed by western analysis (Figure 3B).

**Figure 3:** OA-NO_2_-induced HIF-1α is dependent on HO-1. **A**) HUVECs were treated with 1 µM ZnBG for 30 min followed by incubation with OA-NO_2_ for the indicated times. AMPK protein and phosphorylation levels and HIF-1α protein expression were assayed as described in Materials and Methods. The blot is representative of three blots obtained from three independent experiments. **B**) HUVECs were incubated with HO-1-specific siRNA or control siRNA for 48 h and then treated with OA-NO_2_ or vehicle for 16 h. After treatment, cell lysates were analyzed for HIF-1α and HO-1 protein levels and AMPK phosphorylation at Thr172. *Lower panels*: summary data (*p<0.05 *vs.* control; ^#^ *p*<0.05 *vs.* OA-NO_2_ group; *n* = 3).

### ERK1/2 is partially responsible for OA-NO_2_/HO-1-mediated HIF-1α induction

Clearly, the HIF pathway plays an important role in the regulation of metabolism under hypoxic conditions; however, a variety of HIF-1 stimuli function independently of oxygen concentration. These stimuli are primarily mediated by proteins that regulate HIF-1 translation. This pathway contrasts with hypoxic stimuli, which act upon pre-existing α-subunits [20]. HIF-1α activation by non-hypoxic stimuli has been linked primarily to the phosphatidylinositol 3-kinase (PI3-K)/Akt pathway and the mitogen-activated protein kinase (MAPK) pathway [22]. Both kinase pathways are known to be intimately associated with the regulation of HIF-1α protein translation, stabilization, and transcriptional activity [23]. Our data indicate that OA-NO_2_ did not activate PI3-K/Akt (data not shown). To determine whether OA-NO_2_-mediated HIF-1α induction is dependent on the MAPK pathway, we examined p38 MAPK and extracellular signal-regulated kinase 1/2 (ERK1/2) phosphorylation following stimulation with OA-NO_2_. Treatment with OA-NO_2_ induced a dose-dependent increase in the phosphorylation of ERK1/2 and p38 MAPK (Figure 4A). ZnBG inhibited OA-NO_2_-induced activation of ERK1/2, suggesting a role for HO-1 in this activation (Figure 4B).

**Figure 4:** OA-NO_2_-induced HIF-1α is partially dependent on ERK1/2. **A**) BAECs were incubated with the indicated concentrations of OA-NO_2_ for 16 h. Protein expression and phosphorylation of p38 MAPK and ERK1/2 were assayed as described in Materials and Methods. The blot is representative of three blots obtained from three independent experiments. **B**) BAECs were treated with ZnBG (1 µM) for 30 min followed by incubation with OA-NO_2_ for 16 h. ERK1/2 phosphorylation levels were monitored by immunoblot analysis, and band density was normalized to total ERK1/2 levels (*lower panel*). The blot is representative of three blots obtained from three independent experiments. *p<0.05 *vs.* control; ^#^ *p*<0.05 *vs.* OA-NO_2_ group. **C**) BAECs were treated with OA-NO_2_ alone or with the ERK1/2 signaling inhibitors, UO126 (10 µM) or PD98059 (50 µM), 1 h before the addition of OA-NO_2_. HIF-1α protein levels were monitored by immunoblot analysis, and band density was normalized to β-actin levels (*lower panel*). The blot is representative of three blots obtained from three independent experiments. *p<0.05 *vs.* control; ^#^ *p*<0.05 *vs.* OA-NO_2_ group.

We next determined whether ERK1/2 was a potential upstream mediator of OA-NO_2_-induced HIF-1α upregulation using the ERK1/2 inhibitor, UO126 (10 µM), and the MAPK/ERK kinase (MEK)-specific inhibitor PD98059 (50 µM). Pre-treatment of BAECs with UO126 or PD98059 decreased HIF-1α levels by approximately 50% relative to cells treated with OA-NO_2_ alone (Figure 4C), suggesting that OA-NO_2_-mediated HIF-1α induction is due, at least in part, to MEK/ERK1/2 activity. UO126 and PD98059 did not affect basal HIF-1α expression. In addition to increasing HIF-1α expression, ERK1/2 has previously been reported to phosphorylate HIF-1α *in vitro*, and this post-translational modification can increase HIF-1α activity, presumably by impeding proteasome/von-Hippel-Lindau (VHL) recognition [20]. Although very little is known about the phosphorylation of HIF-1α, this phosphorylation event may be important for optimal activity of the HIF-1 pathway.

### HIF-1α induction by OA-NO_2_ contributes to intracellular Ca^2+^ accumulation and AMPK activation

To examine the involvement of the HIF-1α pathway in OA-NO_2_-mediated AMPK activation, we employed the widely used HIF-1α inhibitor, 3-(5′-hydroxymethyl-2′-furyl)-1-benzylindazole (YC-1) and HIF-1α siRNA. Pre-treatment of BAECs with YC-1 or HIF-1α siRNA significantly inhibited the OA-NO_2_-induced increase in AMPK Thr172 phosphorylation levels relative to OA-NO_2_ treatment alone (Figure 5A and B). Since OA-NO_2_-induced AMPK activation is LKB1-independent, we postulated that the Ca^2+^/CaMKK pathway plays a role in the activation of AMPK by OA-NO_2_/HIF-1α. In addition, because HIF-1α has been reported to regulate Ca^2+^ homeostasis in pulmonary arterial smooth muscle cells via upregulation of store-operated Ca^2+^ channels and enhanced Ca^2+^ influx [24], we examined a possible role for HIF-1α in this process. To determine whether OA-NO_2_ affected endothelial cell [Ca^2+^]_i_, we measured intracellular fluorescence in Fluo-4–loaded BAECs. We found that OA-NO_2_ treatment produced an approximately 1.4- to 2.2-fold increase in [Ca^2+^]_i_ at 6 and 16 h after treatment, respectively (Figure 5C). To confirm a role for HIF-1α in this OA-NO_2_-mediated [Ca^2+^]_i_ increase, we used pharmaceutical- and genetic-inhibition strategies to downregulate HIF-1α. Pre-treatment of BAECs with YC-1 or transfection of these cells with HIF-1α siRNA partially suppressed the OA-NO_2_-induced increases in [Ca^2+^]_i_ (Figure 5D), indicating that this process is at least partially dependent on HIF-1α. We further investigated whether a Ca^2+^ signal is involved in OA-NO_2_-induced AMPK activation using BAPTA-AM, a cell-permeable Ca^2+^ chelator that is widely used as an intracellular Ca^2+^ “sponge”. Our results indicate that chelation of intracellular Ca^2+^ by BAPTA-AM (25 µM, 30 min) significantly inhibited OA-NO_2_-stimulated AMPK phosphorylation (∼60%, *p*<0.05; Figure 5E). Together, these data show that intracellular Ca^2+^ is necessary for OA-NO_2_-induced AMPK activation.

**Figure 5:** HIF-1α mediates OA-NO_2_-induced intracellular Ca^2+^ accumulation and AMPK activation. **A**) BAECs were treated with YC-1 (30 µM) for 30 min followed by incubation with OA-NO_2_ for the indicated times. AMPK phosphorylation and protein levels were assayed as described in Materials and Methods. The blot is representative of three blots obtained from three independent experiments. **B**) BAECs were incubated with HIF-1α-specific siRNA or control siRNA for 48 h and then treated with OA-NO_2_ or vehicle for 16 h. After treatment, cell lysates were analyzed for HIF-1α and AMPK protein levels and AMPK phosphorylation at Thr172. *Lower panels*: summary data (*p<0.05 *vs.* control; ^#^ *p*<0.05 *vs.* OA-NO_2_ group; *n* = 3). **C**) BAECs were incubated with OA-NO_2_ (2.5 µM) for the indicated times. Intracellular Ca^2+^ was measured with Fluo-4 fluorescent dye as described in Materials and Methods. *p<0.01 *vs.* control (*n* = 4). **D**) BAECs were pre-treated with YC-1 (30 µM) or BAPT-AM (25 µM) for 30 min or HIF-1α siRNA or control siRNA for 48 h followed by incubation with OA-NO_2_ for 16 h. After treatment, intracellular Ca^2+^ was measured in intact cells using a Fluo-4 NW kit. *p<0.05 *vs.* control; ^#^ *p*<0.05 vs. OA-NO_2_ group (*n* = 3). **E**) BAECs were pre-loaded with 25 µM BAPT-AM for 30 min prior to incubation with 2.5 µM OA-NO_2_ for 16 h. AMPK protein levels and phosphorylation at Thr172 were detected as described above. Representative blots (top) and densitometric analyses (bottom) are shown. Values are means ± SD from three independent measurements. *p<0.05 *vs.* control; ^#^ *p*<0.05 *vs.* OA-NO_2_ group.

### CaMKKβ mediates OA-NO_2_-induced AMPK activation

Both the tumor suppressor LKB1 [14] and CaMKK [15] are important AMPK kinases as each activates AMPK by directly phosphorylating the AMPK α subunit on Thr172. As shown above (Figure 2A–C), LKB1 is unlikely involved in the activation of AMPK by OA-NO_2_. Because treatment with OA-NO_2_ elevated [Ca^2+^]_i_ and OA-NO_2_-stimulated AMPK activation was Ca^2+^ sensitive, we speculate that the AMPK kinase, CaMKKβ, which is activated by Ca^2+^/calmodulin binding, may be involved. To test this hypothesis, we used the relatively selective CaMKKα and CaMKKβ inhibitor, STO-609 (1 µM) [25] and the competitive CaM inhibitor, KN-93 (3 µM). Either STO-609 or KN-93 was sufficient to prevent activation of AMPK by OA-NO_2_ (Figure 6A), suggesting the involvement of CaMKK in this activation. A specific role for CaMKKβ was indicated by the results of siRNA experiments, which showed that downregulation of CaMKKβ caused a significant reduction in OA-NO_2_-stimulated AMPK phosphorylation (Figure 6B). Downregulation of CaMKKβ protein was verified by western blot analysis. These results suggest that CaMKKβ is the major AMPK kinase under these conditions. To further validate this notion, we determined whether treatment with OA-NO_2_ enhanced the association between CaMKK and AMPK as this interaction is a prerequisite for AMPK phosphorylation/activation. Indeed, following OA-NO_2_ treatment, an enhanced CaMKK and AMPK association was detected by immunoprecipitation with either AMPK or CaMKK antibodies (Figure 6C). Moreover, pre-treatment with YC-1 dramatically inhibited the OA-NO_2_-induced increased CaMKK-AMPK association, further substantiating the indispensable role of HIF-1α in OA-NO_2_-induced AMPK activation.

**Figure 6:** CaMKK is the upstream AMPKK that mediates OA-NO_2_-induced AMPK activation. **A**) HUVECs were treated with STO-609 (1 µM) or KN-93 (3 µM) for 1 h followed by incubation with OA-NO_2_ for 16 h. AMPK and eNOS phosphorylation and protein expression were assayed as described in Materials and Methods. The blot is representative of three blots obtained from three independent experiments. *Lower panels*: summary data (*p<0.05 *vs.* control; ^#^ *p*<0.05 *vs.* OA-NO_2_ group; *n* = 3). **B**) HUVECs were incubated with CaMKKβ-specific siRNA or control siRNA for 48 h and then treated with OA-NO_2_ for 16 h. After treatment, cell lysates were analyzed for AMPK and eNOS phosphorylation and protein levels. *Lower panels*: summary data (*p<0.05 *vs.* control; ^#^ *p*<0.05 *vs.* OA-NO_2_ group; *n* = 3). **C**) HUVECs were pre-treated with YC-1 (30 µM) for 30 min followed by incubation with OA-NO_2_ for 16 h. An immunoblot of AMPK precipitated with an anti-CaMKK antibody is shown. The blot is representative of three blots obtained from three independent experiments. *Lower panels*: summary data (*p<0.05 *vs.* control; ^#^ *p*<0.05 *vs.* OA-NO_2_ group; *n* = 3).

### OA-NO_2_-induced eNOS phosphorylation is dependent on AMPK

We previously demonstrated that AMPK phosphorylates and activates eNOS in cultured endothelial cells [26]. Similarly, Zhang *et al.* demonstrated that infection of endothelial cells with a recombinant adenovirus expressing constitutively active AMPK resulted in eNOS activation and increased NO production [27]. Here, we used phosphorylation of Ser1177 in eNOS, which is a reported substrate of AMPK, as an indicator of AMPK activity in this system. As shown in Figure 7A, incubation of BAECs with OA-NO_2_ increased eNOS Ser1177 phosphorylation in a dose-dependent manner that was very similar to that for AMPK phosphorylation. The time course of OA-NO_2_–induced eNOS phosphorylation was also similar to that for AMPK phosphorylation (Figure 7B). To confirm that OA-NO_2_-stimulated eNOS phosphorylation involved AMPK, we infected BAECs with adenovirus encoding a dominant-negative form of AMPK (Ad-DN-AMPK). As expected, phosphorylation of both AMPK and eNOS was increased after treatment of control BAECs (Ad-GFP-infected or non-infected BAECs) with 2.5 µM OA-NO_2_ for 16 h (Figure 7C). In contrast, overexpression of Ad-DN-AMPK completely abolished OA-NO_2_-induced eNOS phosphorylation. Consistent with a role for AMPK in phosphorylating eNOS, treatment with STO-609 or KN-93 to inhibit the AMPK kinase CaMKK or downregulation of CaMKKβ using siRNA prevented OA-NO_2_-induced eNOS phosphorylation (Figure 6A and B).

**Figure 7:** AMPK mediates OA-NO_2_-induced eNOS phosphorylation and NO production in BAECs. BAECs were treated with (**A**) different concentrations of OA-NO_2_ for 16 h or (**B**) 2.5 µmol/L OA-NO_2_ for the indicated times. Lysates were analyzed by western blot for the indicated proteins. The blot is representative of three blots obtained from three separate experiments. **C**) Western blot of phosphorylated AMPK and eNOS in OA-NO_2_-stimulated BAECs infected with Ad-DN-AMPK (MOI = 50). Non-infected cells or cells infected with Ad-GFP served as controls. For **A–C**, the corresponding densitometric analyses are shown. *p<0.05 *vs.* control; ^#^ *p*<0.05 *vs.* GFP with OA-NO_2_-treated group. **D**) NO release by OA-NO_2_-stimulated BAECs infected with Ad-DN-AMPK (MOI = 50) or Ad-GFP (control). *p<0.05 *vs.* non-transfected, no OA-NO_2_ group; ^#^ *p*<0.05 *vs.* OA-NO_2_-treated, Ad-GFP group. **E**) AMPK activity corresponding to **C** and **D** above. *p<0.05 *vs.* no OA-NO_2_ treatment, Ad-GFP group; ^#^ *p*<0.05 *vs.* OA-NO_2_-treated, Ad-GFP group. **F**) The proposed signaling pathway involved in AMPK/eNOS activation in response to OA-NO2 treatment in endothelial cells.

Both Akt and AMPK are capable of phosphorylating eNOS at Ser1179 [28]. Thus, we determined whether Akt also contributes to OA-NO_2_-induced eNOS phosphorylation. OA-NO_2_ did not increase basal Akt phosphorylation of Ser473 (data not shown), suggesting that OA-NO_2_-stimulated eNOS phosphorylation does not require Akt but depends on activation of AMPK.

Next, we determined whether OA-NO_2_-induced eNOS phosphorylation was associated with increased NO release. Treatment with OA-NO_2_ significantly increased NO release, an effect that was inhibited by Ad-DN-AMPK transfection (Figure 7D). Importantly, Ad-DN-AMPK transfection reduced AMPK activity in OA-NO_2_-treated cells to below control levels (Figure 7E). These results indicate that OA-NO2 increases NO release via AMPK activation.

## Discussion

OA-UFAs are unique signaling mediators that are present in a variety of cell types, including endothelial cells [29]. Considerable evidence points to a role for circulating OA-UFAs in vascular-protective effects [9], although the mechanisms by which OA-NO_2_ are incompletely understood. In this study, we report that OA-NO_2_ activates AMPK in endothelial cells via a Ca^2+^-dependent pathway, and we implicate CaMKKβ as the responsible upstream kinase. Our results show that HIF-1α is an inducer of the intracellular Ca^2+^ mobilization that leads to AMPK activation. On the basis of the results of experiments with an HO-inhibitor and HO-1 siRNA, we also implicate HO-1 in OA-NO_2_-induced upregulation of endothelial HIF-1α.

HO is a rate-limiting enzyme in heme degradation and functions to convert heme to biliverdin, carbon monoxide (CO) and iron. Human HO occurs in two main isoforms, the inducible HO-1 form and the constitutive HO-2 form. Previous studies demonstrated that HO-1 exerts anti-inflammatory effects [30], including prolongation of cardiac xenograft graft survival [31] and inhibition of leukocyte transendothelial migration during complement-dependent inflammation [32] and in response to low-density lipoprotein (LDL) oxidation [33]. More importantly, once induced, HO-1 also confers vascular cytoprotection [30]. The importance of this result is demonstrated by the severe and persistent endothelial damage observed in the case of human HO-1 deficiency [34] and in gene-targeted mice deficient in HO-1 [35]. Furthermore, induction of HO-1 may directly regulate endothelial cell activation, preventing adhesion molecule expression and chronic graft rejection [36]. *In vitro*, HO-1 protects endothelial cells from hydrogen peroxide–mediated cell death [37] and from tumor necrosis factor α (TNFα) cytotoxicity [38]. In addition, HO-1 has been suggested to play a role in angiogenesis. This supposition is supported by the observation that overexpression of HO-1 induces proliferation and formation of capillary-like structures [39]. Thus, therapeutic induction of HO-1 may be beneficial in the treatment of chronic inflammatory diseases as well as cardiovascular diseases. Our results indicate that OA-NO_2_ potently induced HO-1 protein expression in endothelial cells. In agreement with our studies, other studies have suggested that HO-1 expression is induced in human aortic endothelial cells (HAECs) by LNO_2_, which shows a higher potency in this context than other established stimuli, including oxidized fatty acids and hemin. This induction of HO-1 expression by NO_2_-FA is not mediated by NO, NF-κB, or PPARγ [40]. A recent study conducted by Liu *et al.* [41] suggested that AMPK activation regulates HO-1 gene expression in endothelial cells via the Nrf2/antioxidant responsive element signaling pathway and that HO-1 contributes to the biological actions of this kinase. Our data do not exclude the possibility that AMPK activation upregulates HO-1 expression at the gene transcription level. As shown in Figure 1E, Ad-DN-AMPK partially blocks OA-NO2-induced HO-1 protein levels, suggesting that AMPK activation may play a small role in HO-1 protein expression; however, OA-NO2 induces HO-1 expression 2.5-fold as early as 4 h after incubation when AMPK is not yet activated (Figure 1B), implying that OA-NO2 induces HO-1 directly or via another unknown pathway. Thus, AMPK does not act upstream of HO-1 production in this system. Current data supports the idea that upregulation of human HO-1 expression by NO_2_-FA requires synergy between the cAMP-dependent response element and the AP-1 sequences in the −4.5 kb HO-1 promoter region [6], [40]; however, the mechanisms involved in these events remain poorly characterized, and the identities of the signaling molecules downstream of HO-1 that mediate the vascular protective effects of nitrated lipids are not entirely known.

The novel finding of this study is that OA-NO_2_ induces HIF-1α expression via HO-1 under non-hypoxic conditions. HIF-1, which exists as a heterodimer composed of the HIF-1α and HIF-1β subunits, has been shown to mediate numerous physiological and pathophysiological responses to hypoxia. Under normoxic conditions, however, HIF-1α is ubiquitinated and rapidly degraded [42] and is thus present at very low levels under these conditions. Under hypoxic conditions, the HIF-1α subunit is induced. Because HIF-1β is constitutively expressed, HIF-1α is responsible for conferring hypoxia sensitivity to heterodimeric HIF-1. Using specific chemical inhibitors, we demonstrated that ERK1/2 partially mediated HO-1–induced HIF-1α expression (Figure 4). In addition to inducing HIF-1α expression, ERK1/2 has been reported to phosphorylate HIF-1α and to thereby increase its activity [20]. The possibility that CO, a metabolite of HO-1 [43], also plays a role in HIF-1α induction by HO-1 cannot be excluded by our data. A recent study by Chin *et al.* [44] suggested that exposure of macrophages to CO resulted in rapid HIF-1α activation and stabilization, which regulates the expression of genes involved in inflammation, metabolism, and cell survival. This previous study also provided evidence that CO may serve as a signaling intermediary between HO-1 and HIF-1α.

Another important find of the present study is that HIF-1α contributes to an increase in [Ca^2+^]_i_, which is responsible for CaMKKβ-dependent AMPK activation (Figure 5 and 6). Pharmaceutical and genetic inhibitors of HIF-1α suppressed OA-NO_2_-induced increases in [Ca^2+^]_i_, suggesting that HIF-1α is involved in the OA-NO2-induced mobilization of Ca^2+^ in endothelial cells. Previous studies demonstrated that hypoxia evokes an increase in [Ca^2+^]_i_ in endothelial cells [45], and presumably, the induction of HIF-1α contributes to this increase in [Ca^2+^]_i_ under hypoxic conditions or under normoxic conditions in the presence of induction factors that activate HIF-1α. The mechanisms that are involved in endothelial Ca^2+^ homeostasis within the vasculature following HIF-1α activation are also largely unknown. Although HIF-1α has been reported to regulate Ca^2+^ homeostasis in pulmonary arterial smooth muscle cells via upregulation of store-operated Ca^2+^ channels and enhanced Ca^2+^ influx [24], the detailed mechanisms remain to be elucidated.

Our results also showed that OA-NO_2_-stimulated AMPK activation was inhibited by chelation of intracellular free Ca^2+^, selective inhibition of CaMKK by STO-609, selective inhibition of Ca^2+^/calmodulin-dependent protein kinase by KN-93, and siRNA-mediated silencing of CaMKK-β expression (Figure 6). In addition, the association between AMPK and CaMKK was enhanced by OA-NO_2_ treatment. Taken together, these data indicate that the HIF-1α/Ca^2+^/CaMKK- pathway is crucial for OA-NO_2_-induced AMPK activation. Furthermore, CaMKK-mediated AMPK activation in endothelium has also recently been reported in response to thrombin [46], adenosine diphosphate (ADP) [47], and bradykinin [48].

Results from previous studies indicated that endothelial AMPK may play an important physiological role in the function of both endothelial cells and the cardiovascular system as a whole; thus, activation of AMPK may provide an explanation for the beneficial effects of OA-NO_2_ on these systems (see review [49]). Our findings show that induction of the CaMKKβ/AMPK pathway by OA-NO_2_ in endothelial cells may have both physiological and therapeutic relevance. First, endothelial AMPK activation by OA-NO_2_ activates nitric oxide synthase (via phosphorylation on Ser 1177) and elevates NO bioavailability, and these effects may not only protect against early events in atherogenesis, such as white cell adherence [50], but may also prevent later steps in atherogenesis, including fibrous plaque formation. Endothelial NO likely represents the most important anti-atherogenic defense molecule in the vasculature [50]. Nitrated lipids act as NO donors *in vitro* and are widely considered to be a possible endogenous source of NO [51]. Enhanced NO production under hyperlipidemic and hypercholesterolemic conditions, such as those that occur with obesity or insulin-resistant status, however, has been associated with low NO bioactivity [52]. Therefore, it is reasonable to postulate that the presence of these nitrated products and the related AMPK/eNOS/NO pathway *in vivo* may actually play a compensatory role, providing an adjustable supply of NO to compensate for the impaired NO bioactivity and endothelial-dependent vasorelaxation that is characteristic of the early steps of vascular disease. Second, AMPK signaling acts as a novel regulator of angiogenesis and is specifically required for endothelial cell migration and differentiation under conditions of hypoxia [53] or in response to adiponectin [54]. Additionally, AMPK-dependent eNOS activity is required for adequate endothelial tube formation [54]. As described above, increased levels of nitrated lipids are formed in the context of the hyperlipidemia associated with obesity and insulin resistance. Thus, the induction of AMPK and angiogenesis by nitrated lipids may also represent an adaptive defense mechanism against impaired angiogenesis and/or vascular injury caused by obesity-related dislipidemia. The role that activated AMPK plays in increasing fatty acid oxidation via phosphorylation and inhibition of ACC and leading to a decrease in the concentration of malonyl-CoA is most important [55]. In addition, AMPK decreases fatty acid incorporation into glycerolipids in some tissues, either secondary to its effect on fatty acid oxidation or via phosphorylation and inhibition of sn-glycerophosphate acyltransferase, the first committed enzyme in diacylglycerol and triglyceride synthesis [56]. Furthermore, endothelial AMPK activity may inhibit glycerol-3-phosphate acyltransferase, which is required for *de novo* synthesis of diacylglycerol [56]. Thus, AMPK may lessen endothelial diacylglycerol production (and thus protein kinase C activation) both by reducing the availability of the FFA substrates required for this synthesis and by directly inhibiting the enzyme that catalyzes it.

In conclusion, we have demonstrated for the first time that NO_2_-UFAs activate AMPK in endothelial cells by a mechanism that depends on an increase in HO-1 followed by HIF-1α protein expression and Ca^2+^/CaMKKβ activation. Our results also indicate that AMPK activity is required for eNOS/NO production in endothelial cells (Figure 7F). The present study further suggests that AMPK activation by nitrated lipids may play an essential role in compensating or protecting vascular endothelial function against vascular injury in obesity-related dyslipidemia. AMPK might be a valid therapeutic target for treating vascular disorders in obesity and type II diabetes.

## Materials and Methods

### Materials

BAECs and cell culture media were obtained from Clonetics Inc. (Walkersville, MD). HUVECs and cell culture media were purchased from Cascade Biologics (Portland, OR). FFA-free bovine serum albumin (BSA) and oleic acid were obtained from Sigma (St. Louis, MO). ZnBG was purchased from Porphyrin Products, Inc. (Logan, UT). OA-NO_2_ was obtained from Cayman Chemical (Ann Arbor, MI), and AICAR was purchased from Toronto Research Chemicals (Toronto, Canada). The MEK inhibitors PD 98059 and UO 126 were obtained from Calbiochem (La Jolla, CA). 3-(5′-hydroxymethyl-2′-furyl)-1-benzylindazole (YC-1) was purchased from AG Scientific Inc. (San Diego, CA). Antibodies against phospho-ACC (Ser79), phospho-AMPK (Thr172), AMPK, phospho-LKB1 (Ser428), LKB1, and phospho-eNOS (Ser1177) were purchased from Cell Signaling (Beverly, MA). The antibodies against ACC were obtained from Alpha Diagnostic International (San Antonio, TX). All other chemicals and organic solvents were of the highest grade and were obtained from Sigma.

### Cell culture and adenoviral infection

BAECs were grown in EBM supplemented with 2% fetal bovine serum and growth factors. HUVECs were maintained in Medium 200 supplemented with a low-serum growth supplement before use. All culture media were supplemented with both penicillin (100 U/ml) and streptomycin (100 µg/ml). Cells between passages 5 and 10 were used for all experiments. All cells were incubated in a humidified atmosphere of 5% CO_2_/95% air at 37°C. BAECs were infected with adenovirus encoding a dominant-negative mutant form of AMPKα (Ad-DN-AMPK) or green fluorescence protein (Ad-GFP) as a control. Infections were performed in 80% confluent cultures of BAECs in media containing 0.1% fetal bovine serum and recombinant adenovirus at the indicated multiplicity of infection (MOI). Cultures were incubated with adenoviruses for 48 h before experimentation. Using these conditions, infection efficiency was typically at least 80%, as determined by GFP expression.

### SiRNA-mediated gene silencing in endothelial cells

HUVECs or BAECs were transfected with LKB1 siRNA, HO-1 siRNA, HIF–1α siRNA, CaMKKβ, or the corresponding scrambled siRNA (negative control) for 48 h using Lipofectamine™ 2000 (Invitrogen) according to the manufacturer's instructions. Infected cells were starved in serum-free medium for 6 h, then exposed to the indicated concentrations of OA-NO_2_ or vehicle for 24 h.

### Measurement of NO production

For NO detection, BAECs grown in 24-well plates were incubated for 30 min in the presence of 15 µM 4,5-diaminofluorescein diacetate (DAF-2 DA) in PBS or in PBS alone (control) in the dark at 37°C. Cells were then washed with PBS to remove excess DAF-2 DA, and the change in fluorescence over 15 min was measured with excitation and emission wavelengths of 485 and 530 nM, respectively, at room temperature using a microplate reader (FL 600, Bio-Tek). Changes in fluorescence were also visualized with a fluorescence microscope (Olympus IX71), and images were captured for analysis [57].

### Measurement of intracellular Ca^2+^

[Ca^2+^]_i_ was measured using a Fluo-4 NW kit from Invitrogen according to the manufacturer's instructions. In brief, BAECs were treated with OA-NO_2_, control or HIF-1α siRNA, YC-1, or BAPTA-AM. The culture medium was then aspirated, cells were washed once with Hepes buffer (pH 7.4), and 1 ml of Hepes buffer with fluorescent dye was added to the cells. After the cells were incubated for 30 min, the fluorescence intensity was measured with excitation and emission wavelengths of 485 and 520 nM, respectively.

### Western blot analysis

BAECs, HUVECs, or Hela-S3 cells were lysed in cold RIPA buffer. Protein concentrations were determined using a bicinchoninic acid protein assay system (Pierce, Rockford, IL). Proteins were analyzed by western blotting with ECL-Plus detection as described previously [58]. Relative PPARγ protein expression was measured in HUVEC nuclear extracts as previously detailed [59].

### AMPK activity assay

AMPK activity was assayed in the presence and absence of AMP (200 µM) using the SAMS peptide, as previously described [60]. AMPK activity was calculated by determining the difference in activity between both conditions.

### Statistical analysis

Statistical comparisons of vasodilation were performed using a two-way analysis of variance (ANOVA), and intergroup differences were analyzed using Bonferroni's post-hoc test. Time-course studies were analyzed using a repeated-measure ANOVA. All other results were analyzed using a one-way ANOVA. Values are expressed as mean ± SD. *P*-values less than 0.05 were considered significant.

## References

[1] Ischiropoulos H, Beckman JS (2003). Oxidative stress and nitration in neurodegeneration: cause, effect, or association?. J Clin Invest.

[2] Zou MH, Cohen R, Ullrich V (2004). Peroxynitrite and vascular endothelial dysfunction in diabetes mellitus.. Endothelium.

[3] Radi R (2004). Nitric oxide, oxidants, and protein tyrosine nitration.. Proc Natl Acad Sci U S A.

[4] Baker PR, Lin Y, Schopfer FJ, Woodcock SR, Groeger AL (2005). Fatty acid transduction of nitric oxide signaling: multiple nitrated unsaturated fatty acid derivatives exist in human blood and urine and serve as endogenous peroxisome proliferator-activated receptor ligands.. J Biol Chem.

[5] Villacorta L, Zhang J, Garcia-Barrio MT, Chen XL, Freeman BA (2007). Nitro-linoleic acid inhibits vascular smooth muscle cell proliferation via the Keap1/Nrf2 signaling pathway.. Am J Physiol Heart Circ Physiol.

[6] Freeman BA, Baker PR, Schopfer FJ, Woodcock SR, Napolitano A (2008). Nitro-fatty acid formation and signaling.. J Biol Chem.

[7] Lima ES, Di Mascio P, Rubbo H, Abdalla DS (2002). Characterization of linoleic acid nitration in human blood plasma by mass spectrometry.. Biochemistry.

[8] Halliwell B (2000). Lipid peroxidation, antioxidants and cardiovascular disease: how should we move forward?. Cardiovasc Res.

[9] Lima ES, Di Mascio P, Abdalla DS (2003). Cholesteryl nitrolinoleate, a nitrated lipid present in human blood plasma and lipoproteins.. J Lipid Res.

[10] Hayashi K, Noguchi N, Niki E (1995). Action of nitric oxide as an antioxidant against oxidation of soybean phosphatidylcholine liposomal membranes.. FEBS Lett.

[11] Kemp BE, Stapleton D, Campbell DJ, Chen ZP, Murthy S (2003). AMP-activated protein kinase, super metabolic regulator.. Biochem Soc Trans.

[12] Kahn BB, Alquier T, Carling D, Hardie DG (2005). AMP-activated protein kinase: ancient energy gauge provides clues to modern understanding of metabolism.. Cell Metab.

[13] Hawley SA, Selbert MA, Goldstein EG, Edelman AM, Carling D (1995). 5′-AMP activates the AMP-activated protein kinase cascade, and Ca2+/calmodulin activates the calmodulin-dependent protein kinase I cascade, via three independent mechanisms.. J Biol Chem.

[14] Hawley SA, Boudeau J, Reid JL, Mustard KJ, Udd L (2003). Complexes between the LKB1 tumor suppressor, STRAD alpha/beta and MO25 alpha/beta are upstream kinases in the AMP-activated protein kinase cascade.. J Biol.

[15] Hurley RL, Anderson KA, Franzone JM, Kemp BE, Means AR (2005). The Ca2+/calmodulin-dependent protein kinase kinases are AMP-activated protein kinase kinases.. J Biol Chem.

[16] Zou MH, Wu Y (2008). AMP-activated protein kinase activation as a strategy for protecting vascular endothelial function.. Clin Exp Pharmacol Physiol.

[17] Hattori Y, Suzuki K, Hattori S, Kasai K (2006). Metformin inhibits cytokine-induced nuclear factor kappaB activation via AMP-activated protein kinase activation in vascular endothelial cells.. Hypertension.

[18] Hawley SA, Davison M, Woods A, Davies SP, Beri RK (1996). Characterization of the AMP-activated protein kinase kinase from rat liver and identification of threonine 172 as the major site at which it phosphorylates AMP-activated protein kinase.. J Biol Chem.

[19] Woods A, Johnstone SR, Dickerson K, Leiper FC, Fryer LG (2003). LKB1 is the upstream kinase in the AMP-activated protein kinase cascade.. Curr Biol.

[20] Ziello JE, Jovin IS, Huang Y (2007). Hypoxia-Inducible Factor (HIF)-1 regulatory pathway and its potential for therapeutic intervention in malignancy and ischemia.. Yale J Biol Med.

[21] Taylor CT (2008). Mitochondria and cellular oxygen sensing in the HIF pathway.. Biochem J.

[22] Wenger RH (2002). Cellular adaptation to hypoxia: O2-sensing protein hydroxylases, hypoxia-inducible transcription factors, and O2-regulated gene expression.. Faseb J.

[23] Brahimi-Horn C, Mazure N, Pouyssegur J (2005). Signalling via the hypoxia-inducible factor-1alpha requires multiple posttranslational modifications.. Cell Signal.

[24] Wang J, Semenza G, Sylvester JT, Shimoda LA (2005). HIF-1 regulates hypoxic-induction of canonical transient receptor potential (TRPC) channels in pulmonary arterial smooth muscle cells.. Faseb J.

[25] Hawley SA, Pan DA, Mustard KJ, Ross L, Bain J (2005). Calmodulin-dependent protein kinase kinase-beta is an alternative upstream kinase for AMP-activated protein kinase.. Cell Metab.

[26] Zou MH, Hou XY, Shi CM, Nagata D, Walsh K (2002). Modulation by peroxynitrite of Akt- and AMP-activated kinase-dependent Ser1179 phosphorylation of endothelial nitric oxide synthase.. J Biol Chem.

[27] Zhang Y, Lee TS, Kolb EM, Sun K, Lu X (2006). AMP-activated protein kinase is involved in endothelial NO synthase activation in response to shear stress.. Arterioscler Thromb Vasc Biol.

[28] Dimmeler S, Fleming I, Fisslthaler B, Hermann C, Busse R (1999). Activation of nitric oxide synthase in endothelial cells by Akt-dependent phosphorylation.. Nature.

[29] Coles B, Bloodsworth A, Clark SR, Lewis MJ, Cross AR (2002). Nitrolinoleate inhibits superoxide generation, degranulation, and integrin expression by human neutrophils: novel antiinflammatory properties of nitric oxide-derived reactive species in vascular cells.. Circ Res.

[30] Bussolati B, Ahmed A, Pemberton H, Landis RC, Di Carlo F (2004). Bifunctional role for VEGF-induced heme oxygenase-1 in vivo: induction of angiogenesis and inhibition of leukocytic infiltration.. Blood.

[31] Soares MP, Lin Y, Anrather J, Csizmadia E, Takigami K (1998). Expression of heme oxygenase-1 can determine cardiac xenograft survival.. Nat Med.

[32] Willis D, Moore AR, Frederick R, Willoughby DA (1996). Heme oxygenase: a novel target for the modulation of the inflammatory response.. Nat Med.

[33] Ishikawa K, Navab M, Leitinger N, Fogelman AM, Lusis AJ (1997). Induction of heme oxygenase-1 inhibits the monocyte transmigration induced by mildly oxidized LDL.. J Clin Invest.

[34] Yachie A, Niida Y, Wada T, Igarashi N, Kaneda H (1999). Oxidative stress causes enhanced endothelial cell injury in human heme oxygenase-1 deficiency.. J Clin Invest.

[35] Poss KD, Tonegawa S (1997). Heme oxygenase 1 is required for mammalian iron reutilization.. Proc Natl Acad Sci U S A.

[36] Soares MP, Brouard S, Smith RN, Bach FH (2001). Heme oxygenase-1, a protective gene that prevents the rejection of transplanted organs.. Immunol Rev.

[37] Motterlini R, Foresti R, Intaglietta M, Winslow RM (1996). NO-mediated activation of heme oxygenase: endogenous cytoprotection against oxidative stress to endothelium.. Am J Physiol.

[38] Polte T, Oberle S, Schroder H (1997). The nitric oxide donor SIN-1 protects endothelial cells from tumor necrosis factor-alpha-mediated cytotoxicity: possible role for cyclic GMP and heme oxygenase.. J Mol Cell Cardiol.

[39] Deramaudt BM, Braunstein S, Remy P, Abraham NG (1998). Gene transfer of human heme oxygenase into coronary endothelial cells potentially promotes angiogenesis.. J Cell Biochem.

[40] Wright MM, Schopfer FJ, Baker PR, Vidyasagar V, Powell P (2006). Fatty acid transduction of nitric oxide signaling: nitrolinoleic acid potently activates endothelial heme oxygenase 1 expression.. Proc Natl Acad Sci U S A.

[41] Liu XM, Peyton KJ, Shebib AR, Wang H, Korthuis RJ (2011). Activation of AMPK stimulates heme oxygenase-1 gene expression and human endothelial cell survival.. Am J Physiol Heart Circ Physiol.

[42] Sutter CH, Laughner E, Semenza GL (2000). Hypoxia-inducible factor 1alpha protein expression is controlled by oxygen-regulated ubiquitination that is disrupted by deletions and missense mutations.. Proc Natl Acad Sci U S A.

[43] Dulak J, Deshane J, Jozkowicz A, Agarwal A (2008). Heme oxygenase-1 and carbon monoxide in vascular pathobiology: focus on angiogenesis.. Circulation.

[44] Chin BY, Jiang G, Wegiel B, Wang HJ, Macdonald T (2007). Hypoxia-inducible factor 1alpha stabilization by carbon monoxide results in cytoprotective preconditioning.. Proc Natl Acad Sci U S A.

[45] Aley PK, Porter KE, Boyle JP, Kemp PJ, Peers C (2005). Hypoxic modulation of Ca2+ signaling in human venous endothelial cells. Multiple roles for reactive oxygen species.. J Biol Chem.

[46] Stahmann N, Woods A, Carling D, Heller R (2006). Thrombin activates AMP-activated protein kinase in endothelial cells via a pathway involving Ca2+/calmodulin-dependent protein kinase kinase beta.. Mol Cell Biol.

[47] da Silva CG, Jarzyna R, Specht A, Kaczmarek E (2006). Extracellular nucleotides and adenosine independently activate AMP-activated protein kinase in endothelial cells: involvement of P2 receptors and adenosine transporters.. Circ Res.

[48] Mount PF, Lane N, Venkatesan S, Steinberg GR, Fraser SA (2008). Bradykinin stimulates endothelial cell fatty acid oxidation by CaMKK-dependent activation of AMPK.. Atherosclerosis.

[49] Zou MH, Wu Y (2008). AMP-activated protein kinase activation as a strategy for protecting vascular endothelial function.. Clin Exp Pharmacol Physiol.

[50] Forstermann U, Munzel T (2006). Endothelial nitric oxide synthase in vascular disease: from marvel to menace.. Circulation.

[51] Gorczynski MJ, Huang J, King SB (2006). Regio- and stereospecific syntheses and nitric oxide donor properties of (E)-9- and (E)-10-nitrooctadec-9-enoic acids.. Org Lett.

[52] Moriel P, Pereira IR, Bertolami MC, Abdalla DS (2001). Is ceruloplasmin an important catalyst for S-nitrosothiol generation in hypercholesterolemia?. Free Radic Biol Med.

[53] Nagata D, Mogi M, Walsh K (2003). AMP-activated protein kinase (AMPK) signaling in endothelial cells is essential for angiogenesis in response to hypoxic stress.. J Biol Chem.

[54] Ouchi N, Kobayashi H, Kihara S, Kumada M, Sato K (2004). Adiponectin stimulates angiogenesis by promoting cross-talk between AMP-activated protein kinase and Akt signaling in endothelial cells.. J Biol Chem.

[55] Ruderman NB, Cacicedo JM, Itani S, Yagihashi N, Saha AK (2003). Malonyl-CoA and AMP-activated protein kinase (AMPK): possible links between insulin resistance in muscle and early endothelial cell damage in diabetes.. Biochem Soc Trans.

[56] Park H, Kaushik VK, Constant S, Prentki M, Przybytkowski E (2002). Coordinate regulation of malonyl-CoA decarboxylase, sn-glycerol-3-phosphate acyltransferase, and acetyl-CoA carboxylase by AMP-activated protein kinase in rat tissues in response to exercise.. J Biol Chem.

[57] Lassegue B, Sorescu D, Szocs K, Yin Q, Akers M (2001). Novel gp91(phox) homologues in vascular smooth muscle cells : nox1 mediates angiotensin II-induced superoxide formation and redox-sensitive signaling pathways.. Circ Res.

[58] Davis BJ, Xie Z, Viollet B, Zou MH (2006). Activation of the AMP-activated kinase by antidiabetes drug metformin stimulates nitric oxide synthesis in vivo by promoting the association of heat shock protein 90 and endothelial nitric oxide synthase.. Diabetes.

[59] Marx N, Bourcier T, Sukhova GK, Libby P, Plutzky J (1999). PPARgamma activation in human endothelial cells increases plasminogen activator inhibitor type-1 expression: PPARgamma as a potential mediator in vascular disease.. Arterioscler Thromb Vasc Biol.

[60] Zou MH, Kirkpatrick SS, Davis BJ, Nelson JS, Wiles WGt (2004). Activation of the AMP-activated protein kinase by the anti-diabetic drug metformin in vivo. Role of mitochondrial reactive nitrogen species.. J Biol Chem.

